The article "Nomogram for preoperative estimation of long-term survival of patients who underwent curative resection with hepatocellular carcinoma beyond Barcelona clinic liver cancer stage A1" was published in 2016. Journal: Oncotarget.

# Nomogram for preoperative estimation of long-term survival of patients who underwent curative resection with hepatocellular carcinoma beyond Barcelona clinic liver cancer stage A1

**DOI:** 10.18632/oncotarget.11358

**Published:** 2016-08-17

**Authors:** Dan-Yun Ruan, Ze-Xiao Lin, Tian-Tian Wang, Hui Zhao, Dong-Hao Wu, Jie Chen, Min Dong, Qu Lin, Xiang-Yuan Wu, Yang Li

**Affiliations:** ^1^ Department of Medical Oncology, The Third Affiliated Hospital of Sun Yat-Sen University, Guangdong, China; ^2^ Department of Liver Surgery, The Third Affiliated Hospital of Sun Yat-Sen University, Guangzhou, China

**Keywords:** hepatocellular carcinoma, Barcelona clinic liver cancer stage, resection, nomogram, survival

## Abstract

**Background and Aims:**

This retrospective cohort study developed a prognostic nomogram to predict the survival of hepatocellular carcinoma (HCC) patients diagnosed as beyond Barcelona clinic liver cancer stage A1 after resection and evaluated the possibility of using the nomogram as a treatment algorithm reference.

**Results:**

The predictors included in the nomogram were total tumour volume, Child-Turcotte-Pugh class, plasma fibrinogen and portal vein tumour thrombus. Patients diagnosed as beyond A1 were stratified into low-, medium- and high-risk groups using nomogram scores of 0 and 51 with the total points of 225. Patients within A1 exhibited similar recurrence-free survival (RFS) and overall survival (OS) rates compared with the low-risk group. Patients in the medium-risk group exhibited a similar OS but a worse RFS rates compared with patients within A1. The high-risk group was associated with worse RFS and OS rates compared with the patients within A1 (3-year RFS rates, 27.0% vs. 60.3%, *P* < 0.001; 3-year OS rates, 49.2% vs. 83.1%, *P* < 0.001).

**Methods:**

A total of 352 HCC patients undergoing curative resection from September 2003 to December 2012 were included to develop a nomogram to predict overall survival after resection. Univariate and multivariate survival analysis were used to identify prognostic factors. A visually orientated nomogram was constructed using a Cox proportional hazards model.

**Conclusions:**

This user-friendly nomogram offers an individualized preoperative recurrence risk estimation and stratification for HCC patients beyond A1 undergoing resection. Resection should be considered the first-line treatment for low-risk patients.

## INTRODUCTION

Hepatocellular carcinoma (HCC) is a lethal tumour with a prognosis that largely depends on the tumour stage at diagnosis and patient access to radical treatment. Western and Eastern groups validated and approved the Barcelona Clinic Liver Cancer (BCLC) staging system as a guide for HCC treatment algorithms [1–3]. The BCLC classification indicates that liver resection should be performed only in patients with a small single HCC nodule without signs of portal hypertension or hyperbilirubinemia [4]. However, improvements in surgical techniques, radiological assessment, patient selection and perioperative management have greatly improved the resectability of tumours and the safety of surgical resections. Portal hypertension is no longer considered a contraindication to liver resection because of the low rates of postoperative mortality and morbidity [5, 6]. Nevertheless, more than 20% of HCC patients with large tumours, even those accompanied by macrovascular invasion, are treated using surgical resection. Resection of HCC is currently possible in 60% of patients in Asia, and 25% to 40% of patients in Western countries [7, 8]. More than half of the patients undergoing curative resection were beyond BCLC stage A [9]. Recent studies have reported that surgical resection may improve long-term survival compared with transarterial chemoembolization (TACE) in intermittent and advanced HCC [10, 11]. However, based on the BCLC classification, HCC patients with multiple nodules, large tumours or macrovascular invasion are recommended palliative treatments, which have unsatisfactory long terms results, instead of surgical treatments even if the lesion is resectable [12, 13]. The BCLC classification has been criticized because it excludes patients who may benefit from curative resection. Debate continues regarding the selection of surgical resection as a first-line treatment for HCC diagnosed as beyond BCLC A1, and the choice is difficult because robust evidence to guide decision-making is still lacking.

The article "Nomogram for preoperative estimation of long-term survival of patients who underwent curative resection with hepatocellular carcinoma beyond Barcelona clinic liver cancer stage A1" was published in 2016. Journal: Oncotarget.

Nomograms are graphical representations of statistical predictive models that generate numerical probabilities of an event, and these models have been applied for various malignancies [14–16]. The ability of nomograms to generate personalized predictions allows their use in patient counselling and risk stratification. Nomograms have been applied to predict recurrence, survival, and distant metastasis after various treatments for HCC [17–19]. To our knowledge, a predictive nomogram for HCC survival beyond BCLC A1 after resection has not been reported. We constructed a simple and clinically relevant nomogram to predict overall survival (OS) in patients beyond BCLC A1 who were undergoing curative resection. We also explored the possibility of using the nomogram for risk stratification and as a treatment reference by comparing recurrence-free survival (RFS) and overall survival in HCC patients in or beyond BCLC A1.

The article "Nomogram for preoperative estimation of long-term survival of patients who underwent curative resection with hepatocellular carcinoma beyond Barcelona clinic liver cancer stage A1" was published in 2016. Journal: Oncotarget.

## RESULTS

### Characteristics of HCC patients undergoing curative surgical resection

A total of 352 HCC patients undergoing curative surgical resection were included in this study. Of these patients, 136 (38.6%) patients were in BCLC stage 0 and A1, and 216 (61.4%) patients were beyond A1. Table 1 summarizes the characteristics of the patients. Most of the patients were men (*n* = 315, 89.5%). Most patients (*n* = 301, 85.8%) were positive for HBsAg and hepatic cirrhosis was present in 69.3% (*n* = 244) of the patients. The median follow-up duration for patients within and beyond A1 was 48 and 42 months, respectively. A total of 201 (57.1%) patients experienced tumour recurrence, mostly within the first 3 years (*n* = 174, 86.6%). A total of 252 patients were alive during follow up. Patients beyond stage A1 exhibited significantly worse RFS and OS compared with patients within stage A1 (*P* < 0.05). The observed 3- and 5-year RFS rates were 60.3% and 55.9%, respectively, for patients within A1 and 44.4% and 37.0%, respectively, for patients beyond A1 (*P* < 0.001). The 3- and 5-year OS rates were 83.1% and 80.1% vs. 76.4% and 70.8%, respectively (*P* < 0.05) (Figure 1A, 1B).

**Table 1:** Baseline demographics of HCC patients receiving curative resection

Variables	Total (*n* = 352)
Age (y, mean ± SD)	50.6 ± 11.7
Male, *n* (%)	315 (89.5)
Drinking, *n* (%)	79 (22.4)
Smoking, *n* (%)	115 (32.7)
HBsAg (+), *n* (%)	301 (85.8)
HCV-IgG (+), *n* (%)	11 (3.1)
HBV DNA copies >1^*^10^4^, *n* (%)	141 (40.1)
Hepatic cirrhosis, *n* (%)	244 (69.3)
Portal hypertension, *n* (%)	152 (43.2)
NLR (mean ± SD)	2.34 ± 1.98
LMR (mean ± SD)	4.73 ± 3.04
PLR (mean ± SD)	108.03 ± 65.46
Fib (g/L, mean ± SD)	3.4 ± 2.0
CTP class A, *n* (%)	296 (84.1)
AFP > 400 ng/mL, *n* (%)	120 (34.1)
Total tumour volume (cm^3^, mean ± SD)	157.7 ± 360.4
Single tumour lesions, *n* (%)	304 (53.7)
Vascular invasion, *n* (%)	73 (20.7)
PVTT, *n* (%)	16 (4.5)
BCLC stage	
Stage 0, *n* (%)	15 (4.2)
Stage A1, *n* (%)	121 (34.4)
Stage A2, *n* (%)	101 (28.7)
Stage A3, *n* (%)	10 (2.8)
Stage A4, *n* (%)	10 (2.8)
Stage B, *n* (%)	22 (6.3)
Stage C, *n* (%)	73 (20.7)

**Figure 1:** (**A**) Overall survival (OS) and (**B**) recurrence-free survival (RFS) for hepatocellular carcinoma patients receiving curative resection within and beyond BCLC A1. Patients beyond BCLC A1 were associated with worse OS and RFS compared with patients within A1. The 3- and 5-year OS rates were 83.1% and 80.1% vs. 76.4% and 70.8%, respectively, *P* < 0.05. The 3- and 5-year RFS rates were 60.3% and 55.9% vs. 44.4% and 37.0%, respectively, *P* < 0.001.

### Construction and validation of the nomogram

Candidate predictors of OS in patients beyond BCLC stage A1 were included in survival analyses. These factors included age, sex, drinking history, smoking history, positive HBsAg status, HBV DNA copy number, positive HCV-IgG status, hepatic cirrhosis, portal hypertension, ascites, serum biochemistry, blood test index, serum a-fetoprotein (AFP) level, tumour number, tumour size, macrovascular invasion and portal vein tumour thrombus (PVTT). Serum biochemistries were dichotomized by the normal range and handled as categorical variables. The optimal cut-off value for TTV was determined using a ROC analysis and was 113 cm^3^. The same method was used to identify the cut-off values for the neutrophil-lymphocyte rate (NLR), lymphocyte-to-monocyte ratio (LMR), platelet-to-lymphocyte ratio (PLR) and plasma fibrinogen level as 3.07, 3.67, 117.17 and 3.43, respectively. Decisions for variable grouping were made prior to actual modelling. The independent prognostic factors in the final Cox model were TTV (≤ 113 cm^3^ and > 113 cm^3^), Child-Turcotte-Pugh class (A and B), plasma fibrinogen level (≤ 3.43 g/L and >3.43 g/L) and PVTT (Table 2).

The article "Nomogram for preoperative estimation of long-term survival of patients who underwent curative resection with hepatocellular carcinoma beyond Barcelona clinic liver cancer stage A1" was published in 2016. Journal: Oncotarget.

**Table 2:** Multivariate regression results for overall survival in hepatocellular carcinoma patients beyond BCLC A1

Category *n* = 216	3-year OS rate (%)	5-year OS rate (%)	Univariate analysis *p*	Multivariate analysis *p*, HR (95% CI)
Gender				
Male	76.6	70.8	0.895	
Female	75.0	70.8		
Age, years				
< 60	76.0	69.6	0.976	
≥ 60	77.8	75.6		
Drinking				
Yes	77.1	70.8	0.931	
No	76.2	70.8		
Smoking				
Yes	72.6	63.0	0.077	
No	78.3	74.8		
HBsAg				
Positive	76.1	69.7	0.359	
Negative	77.8	77.8		
HBV DNA copies				
> 1*10^4^	76.4	67.4	0.530	
≤ 1*10^4^	76.4	73.2		
HVC-IgG				
Positive	66.7	66.7	0.826	
Negative	76.6	70.8		
Hepatic cirrhosis				
Yes	76.2	69.6	0.500	
No	77.1	75.0		
Portal hypertension				
Yes	76.3	69.1	0.400	
No	76.6	75.0		
CTP class				0.008*
A	79.6	74.3	0.006*	2.128
B	65.3	59.2		(1.213–3.733)
NLR				0.270
> 3.07	58.0	54.0	0.000*	1.467
≤ 3.07	81.9	75.9		(0.743–2.898)
LMR				0.094
> 3.67	84.8	79.5	0.000*	0.619
≤ 3.67	63.1	57.1		(0.353–1.084)
PLR				0.446
> 117.17	62.5	60.9	0.005*	0.774
≤ 117.17	82.2	75.0		(0.400–1.497)
Fib				0.049*
> 3.43 g/L	58.9	56.2	0.000*	1.758
≤ 3.43 g/L	85.3	78.3		(1.001–3.088)
AFP				
> 400 ng/mL	67.5	65.0	0.235	
≤ 400 ng/mL	81.6	74.3		
Total tumour volume				0.017*
> 113 cm^3^	58.3	54.2	0.000*	2.056
≤ 113 cm^3^	85.4	79.2		(1.135–3.724)
Tumour lesions				
Single	75.6	70.2	0.913	
Multiple	79.2	72.9		
Vascular invasion				0.607
Yes	61.6	61.6	0.007*	0.845
No	83.9	75.5		(0.446–1.603)
PVTT				0.000*
Yes	18.8	18.8	0.000*	6.392
No	81.0	75.0		(2.857–14.298)

The nomogram was constructed using β-coefficients from the final Cox multivariate model. PVTT had the highest impact in the model, and it was given 100 points in the nomogram. The nomogram points for other variables were allocated according to the ratios of β-coefficients between PVTT and the selected variables (Figure 2A). The concordance index for the model in predicting overall survival for HCC patients beyond BCLC A1 after curative resection was 0.718, and the 95% CI of the concordance index was 0.786 to 0.651 with bootstrapping (cycle = 100). A calibration curve was plotted at 3-year intervals. The AUC of the nomogram for assessing 3-year OS after resection was 0.775 (95% CI 0.698–0.853, *P* < 0.001, Figure 2B and 2C). For BCLC staging system, the AUC was 0.631.

The article "Nomogram for preoperative estimation of long-term survival of patients who underwent curative resection with hepatocellular carcinoma beyond Barcelona clinic liver cancer stage A1" was published in 2016. Journal: Oncotarget.

**Figure 2:** (**A**) Nomogram predicting overall survival for hepatocellular carcinoma patients beyond BCLC A1 receiving curative resection. To calculate the probability of overall survival, sum up the points identified on the scale for the 4 variables and draw a vertical line from the total points scale to the probability scale. (**B**) Calibration plot of the nomogram. Calibration curves of the nomogram at 3 years showed good correlation between predicted and observed outcomes. The calibration curve was close to the 45-degree line. (**C**) ROC curves of the nomogram for assessing the 3-year OS rate. The AUC was 0.775 (95% CI 0.698–0.853, *P* < 0.001).

### Risk group classification and survival analysis

The first and last one-third values of the nomogram score in patients beyond BCLC A1 were 0 and 51, respectively. Patients were further divided into three subgroups using these two nomogram scores. Patients with nomogram scores = 0 were considered the low-risk group (*n* = 83), and patients with nomogram scores > 51 were considered the high-risk group (*n* = 63). The remaining patients (*n* = 70) were in the medium-risk group (Table 3). Patients in the medium-risk group exhibited worse RFS but similar OS compared with patients in the low-risk group. The 3- and 5-year RFS rates were 41.4% and 35.7% vs. 60.2% and 50.6%, respectively, for the medium-risk group vs. the low-risk group, respectively (*P* < 0.05). The 3- and 5-year OS rates were 82.9% and 78.6% vs. 91.6% and 83.1%, respectively (*P* = 0.253). Patients in the medium-risk group exhibited improved RFS and OS compared with patients in the high-risk group. The 3- and 5-year RFS rates were 41.4% and 35.7% vs. 27.0% and 20.6%, respectively, for the medium-risk group vs. the high-risk group, respectively (*P* < 0.05). The 3- and 5-year OS rates were 82.9% and 78.6% vs. 49.2% and 46.0%, respectively (*P* < 0.001) (Figure 3A and 3B).

**Table 3:** BCLC stages for patients in low, median and high risk groups

BCLC stage	Risk Group Classification of Nomogram		
	Low-risk group	Medium-risk group	High-risk group
Stage A2–A4	67	40	14
Stage B	5	12	5
Stage C	11	18	44

The article "Nomogram for preoperative estimation of long-term survival of patients who underwent curative resection with hepatocellular carcinoma beyond Barcelona clinic liver cancer stage A1" was published in 2016. Journal: Oncotarget.

**Figure 3:** (**A**) OS and (**B**) RFS for hepatocellular carcinoma patients beyond BCLC A1 in the low-, medium- and high-risk groups. Patients in the medium-risk group had similar OS but worse RFS compared with patients in the low-risk group. The 3- and 5-year OS rates were 82.9% and 78.6% vs. 91.6% and 83.1%, respectively, *P* = 0.253; the 3- and 5-year RFS rates were 41.4% and 35.7% vs. 60.2% and 50.6%, respectively, *P* < 0.05. Patients in the medium-risk group had better OS and RFS compared with patients in the low-risk group. The 3- and 5-year OS rates were 82.9% and 78.6% vs. 49.2% and 46.0%, respectively, *P* < 0.001. The 3- and 5-year RFS rates were 41.4% and 35.7% vs. 27.0% and 20.6%, respectively, *P* < 0.01.

The low-risk patients exhibited similar RFS and OS rates compared with patients within BCLC stage A1 (Figure 4A and 4B). The RFS and OS rates of the high-risk group were significantly worse compared with patients within BCLC stage A1 (Figure 6A and 6B). However, patients within BCLC A1 exhibited a similar OS but improved RFS compared with patients in the medium-risk group. The 3- and 5-year RFS rates were 60.3% and 55.9% vs. 41.4% and 35.7%, for the patients within A1 vs. the medium-risk group, respectively (*P* < 0.05). The 3- and 5-year OS rates were 83.1% and 80.1% vs. 82.9% and 78.6%, respectively (*P* = 0.635) (Figure 5A and 5B).

**Figure 4:** (**A**) OS and (**B**) RFS for hepatocellular carcinoma patients within BCLC A1 and the low-risk group. Patients within BCLC A1 had similar OS and RFS compared with patients in the low-risk group. The 3- and 5-year OS rates were 83.1% and 80.1% vs. 91.6% and 83.1%, respectively, *P* = 0.462. The 3- and 5-year RFS rates were 60.3% and 55.9% vs. 60.2% and 50.6%, respectively, *P* = 0.689.

**Figure 5:** (**A**) OS and (**B**) RFS for hepatocellular carcinoma patients within BCLC A1 and the medium-risk group. Patients within BCLC A1 had similar OS but better RFS compared with patients in the medium-risk group. The 3- and 5-year OS rates were 83.1% and 80.1% vs. 82.9% and 78.6%, respectively, *P* = 0.635. The 3- and 5-year RFS rates were 60.3% and 55.9% vs. 41.4% and 35.7%, respectively, *P* < 0.05.

**Figure 6:** (**A**) OS and (**B**) RFS for hepatocellular carcinoma patients within BCLC A1 and the high-risk group. Patients within BCLC A1 had better RFS and OS compared with patients in the high-risk group. The 3- and 5-year OS rates were 83.1% and 80.1% vs. 49.2% and 46.0%, respectively, *P* < 0.001. The 3- and 5-year RFS rates were 60.3% and 55.9% vs. 27.0% and 20.6%, respectively, *P* < 0.001.

The article "Nomogram for preoperative estimation of long-term survival of patients who underwent curative resection with hepatocellular carcinoma beyond Barcelona clinic liver cancer stage A1" was published in 2016. Journal: Oncotarget.

The BCLC B and C patients in low- and median-risk groups exhibited a similar OS which was much better than BCLC B and C patients receiving TACE. The 5-year OS rates were 87.5% and 83.3% vs. 27.5% (*P* < 0.001). The BCLC B and C patients in high-risk group exhibited a similar OS compared with BCLC B and C patients receiving TACE. The 5-year OS rates were 46.9% vs. 27.5% (*P* = 0.079) (Figure 7A and 7B).

**Figure 7:** (**A**) OS for BCLC B/C hepatocellular carcinoma patients in low- and median-risk groups and BCLC B/C patients receiving TACE. The BCLC B/C patients in low- and median-risk groups exhibited a similar OS which was much better than BCLC B/C patients receiving TACE. The 5-year OS rates were 87.5% and 83.3% vs. 27.5% (*P* < 0.001). (**B**) OS for BCLC B/C hepatocellular carcinoma patients in high risk group and BCLC B/C patients receiving TACE. The BCLC B/C patients in high-risk group exhibited a similar OS compared with BCLC B/C patients receiving TACE. The 5-year OS rates were 46.9% vs. 27.5% (*P* = 0.079).

## DISCUSSION

The BCLC classification links stage stratification with corresponding therapeutic recommendations, and liver resection is recommended for patients harbouring solitary tumours and very well-preserved liver function (BCLC stage 0 and A1) [4]. The ratio of patients who received radical resection (60%) was higher in our study compared with the 50% of patients who would not have been recommended surgery but still underwent surgery in Western countries [9]. We found that patients undergoing radical resection within stage A1 were associated with superior overall survival and lower recurrence compared with patients beyond stage A1. A significant number of patients with HCC do not match the therapeutic criteria corresponding to their BCLC stage, but some of these patients may still benefit from surgical treatments that are not recommended by the current guidelines [20]. Patients in the medium-risk group in our study achieved a 5-year overall survival rate of 78.6% after resection, which was comparable to patients within stage A1. A recent meta-analysis demonstrated a statistically significant survival benefit of hepatic resection over TACE in intermediate and advanced stages of disease [21]. Therefore, we aimed to develop a clinically relevant method to predict survival in patients beyond BCLC stage A1.

We constructed a predictive nomogram from a large patient cohort receiving radical resection beyond BCLC A1 that is capable of generating personalized risk estimations for overall survival after surgery. This easy-to-use graphical tool consists of ordinary clinical variables, including total tumour volume, PVTT, CTP classification and plasma fibrinogen level. TTV, as a composite of the maximum diameter and number of tumour nodules, is a feasible prognostic predictor for HCC patients undergoing locoregional therapy [22]. Our data indicated that TTV > 113 cm^3^, which corresponds to a single nodule of 6 cm in maximum diameter, is an independent prognostic predictor of poor survival. Macrovascular invasion is one of the strongest predictors of survival in HCC patients because it is related to an increased risk of intrahepatic or extrahepatic metastases [23, 24]. The 5-year survival rates for selected patients with PVTT ranged from 11% to 42% [25–27]. The 5-year overall survival in our study was 18.8%, with a median survival of 12 months. Notably, patients with macrovascular invasion but PVTT exhibited comparable survival to patients without macrovascular invasion. The underlying disease also primarily causes insufficient liver function. Up to 80% of HCC cases are attributed to chronic HBV infection in China [28]. CTP class B was associated with poor survival and a high recurrence rate in our study, and 86% of these patients were HbsAg-positive. The nomogram consisted of tumour burden, surrogates for underlying liver conditions and indexes that represent the tumour immunomicroenvironment. The interaction of fibrinogen with platelets may protect tumour cells from natural killer cytotoxicity [29]. Fibrinogen deposition around tumour cells enhances the interaction between platelets and tumour cells, which is critical for haematogenous metastasis of the tumour [30]. Our data indicated that elevated plasma fibrinogen remained a significant risk factor for HCC recurrence and overall survival, which is consistent with several previous studies [31, 32]. Patients with plasma fibrinogen levels exceeding 3.43 g/L had lower 3-year OS rates than patients with fibrinogen levels below 3.43 g/L (58.9% and 85.3%, *P* < 0.001). We further divided the patients into 3 distinct risk groups according to the first and last one-third of the nomogram scores. The nomogram exhibited great discriminatory ability between the low, medium and high-risk groups. Notably, the nomogram did not incorporate pathological features, but it was derived solely from pre-treatment clinical variables. These features enable the nomogram to be an integral part of pre-treatment counselling and decision-making.

The article "Nomogram for preoperative estimation of long-term survival of patients who underwent curative resection with hepatocellular carcinoma beyond Barcelona clinic liver cancer stage A1" was published in 2016. Journal: Oncotarget.

Surgery is a good option for patients in the low-risk group not only because of the comparable outcomes of patients within BCLC A1 after resection but the much better prognosis compared with patients receiving TACE. Patients in the medium-risk group should receive intensive follow-up after surgery because of the higher recurrence rate compared with patients in BCLC A1. The results of recent studies supported significantly better survival in patients with intermediate HCC who underwent hepatic resection compared with TACE [13]. Our study showed that the BCLC B and C patients in low and median-risk group exhibited better OS compared with TACE. But for high-risk group, there is no advantage. Our nomogram indicated that patients in the high-risk group were generally accompanied by TTV > 113 cm^3^ and CTP class B. Unsatisfactory therapeutic results are achieved in these patients, and the insufficient volume and function of the liver remnant raises a high risk of postoperative hepatic dysfunction and death. The pros and cons of surgery should be carefully considered for these patients.

There are several important considerations for constructing a nomogram. The numbers of dead and alive patients should be greater than 10 times the number of predictors for OS predictions to reduce the expected error in the predicted probabilities to less than 10% [14]. The model must be validated using data-splitting or resampling with bootstrapping. Data-splitting is commonly used, but it exhibits the disadvantage of reduced accuracy. Resampling with bootstrapping can provide nearly unbiased estimates of model performance without sacrificing the sample size [33]. The number of deaths in this study was 69, which is 17 times greater than the number of predictors used in the nomogram. We also applied the internal validation with resampling method by bootstrapping the entire cohort to calibrate the nomogram. These approaches further increase the validity and data integrity of our results.

This study has some limitations. First, this retrospective study is prone to certain biases that could not be completely avoided. Second, more patients undergoing TACE should be involved for further matching comparisons to confirm the nomogram for improving treatment selection in a randomized control trial. Finally, this study was dependent on a single institutional cohort of patients from the Asia-Pacific region, and the main underlying disease was hepatitis B. Multicentre prospective studies are required to validate the prognostic accuracy determined herein.

In conclusion, we constructed a clinically relevant and easy-to-use nomogram that consistently predicted overall survival after radical resection for HCC patients beyond BCLC stage A1. Investigators may use this nomogram to provide specific information on individual prognosis and classify patients receiving surgical resection into low-, medium- and high-risk groups. We further demonstrated that patients in the low-risk group shared similar OS and RFS rates compared with patients within BCLC A1. Close monitoring after resection is necessary for the medium-risk group because of the worse RFS compared with BCLC stage 0 and A1 patients. However, surgical resection for patients in the high-risk group should be performed only after careful consideration. This nomogram may be a useful reference resource to improve treatment selection for HCC patients beyond BCLC A1. These results require external validation and further justification in adequately designed trials, but our findings support the use of the nomogram for the risk stratification and treatment of low-risk patients with radical resection to achieve an improved prognosis.

The article "Nomogram for preoperative estimation of long-term survival of patients who underwent curative resection with hepatocellular carcinoma beyond Barcelona clinic liver cancer stage A1" was published in 2016. Journal: Oncotarget.

## MATERIALS AND METHODS

### Patient selection and data collection

We retrospectively reviewed the medical records of patients with pathologically diagnosed HCC who underwent curative resection between September 2003 and December 2012 at our institution. The following selection criteria were used: 1) no extrahepatic tumour or lymph node metastasis; 2) no positive surgical margin upon resection; 3) no perioperative period death; 4) newly diagnosed HCC without neoadjuvant therapy; and 5) regular follow up; 6) ECOG 0-1, tolerate operation. 7) The tumour, satellite nodules and involved vascular located within one lobe, or satellite nodules could be removed by local resection. 8) The volume of non-tumour lobe is over 50% of total liver volume. 9) CTP class A, CTP class B reached class A after liver-protecting therapy, CTP class B with normal oral glucose tolerance test. 10) Combined with ultrasound, CT, MRI examination and the appearance of cirrhosit liver during surgery, the resection would be decided finally. A total of 352 HCC patients were included in this study. The study protocol was designed in accordance with the guidelines outlined in the Declaration of Helsinki, and the Ethics Committee of the Third Affiliated Hospital of Sun Yat-sen University approved the protocol. Informed consent was obtained from all patients.

The HCC preoperative diagnosis was based on EASL HCC management guidelines [4]. The total tumour volume was calculated as the sum of the volumes of all tumours to indicate the tumour burden using a standard equation: tumour volume (cm^3^) = 4/3 × 3.14 × r^3^ (*r* = the maximum radius of each measurable tumour nodule). Recurrent tumours were defined as radiological evidence of residual tumours adjacent to the original tumour and residual tumours inside or outside the liver. A follow-up was performed once every 6 months for the first 3 years and every year thereafter. Follow-up consisted of physical examination, routine blood chemistry, serum AFP, chest X-ray, and abdominal ultrasound. Further examinations (PET-CT, CT or MRI) were conducted in cases with suspicious lesions on ultrasound and an elevated AFP to confirm or exclude recurrence.

The article "Nomogram for preoperative estimation of long-term survival of patients who underwent curative resection with hepatocellular carcinoma beyond Barcelona clinic liver cancer stage A1" was published in 2016. Journal: Oncotarget.

### Development, validation, and risk stratification of the nomogram

We used overall survival after surgery as the primary endpoint in this study. Factors that were significant (*P* < 0.05) for the prediction of overall survival in a univariate survival analysis were selected for a multivariate survival model. Confidence intervals (CIs) and hazard ratios (HRs) were calculated. β-coefficients from a final Cox model were used to construct the nomogram.

A 3-step validation of the nomogram was used. First, a Harrell concordance index was used to determine the discriminating ability of the nomogram. An internal validation with 100 sets of full bootstrap samples was performed to evaluate the ability to predict the OS for resection patients. Second, patients were grouped into quartiles of nomogram scores, and a calibration plot was drawn to compare the predicted probabilities of survival with observed survival at 3-year intervals after curative resection. Third, the AUC of the nomogram for assessing 3-year OS after resection was calculated. The first and last one-third values of the nomogram scores were used to stratify patients into 3 groups for further analysis (low-, medium- and high-risk).

To compare the prognosis of patients receiving resection with TACE, 150 patients receiving TACE from October 2010 to December 2012 were collected. 51 patients with resection potential in BCLC B and C were finally involved for further comparison.

### Statistical analysis

Categorical data were evaluated using a chi-square test and Fisher's exact test. A Mann-Whitney *U* test was used for continuous variables. The RFS and OS rates were examined using the Kaplan-Meier method. A receiver operating characteristic (ROC) analysis was performed to determine the cut-off value. All statistical analyses were conducted using SPSS 16.0 for Windows (SPSS Inc., Chicago, IL), MedCalc version 11.4 (The MedCalc software, Mariakerke, Belgium), R 3.1.0 (Lucent Technologies, New Jersey, USA) and SAS version 9.4 for Windows (SAS Institute, Inc., Cary, NC). Statistical significance was set at *P* < 0.05.
